The article "Molecular Hydrogen Effectively Heals Alkali-Injured Cornea via Suppression of Oxidative Stress" was retracted in 2022. Reasons: duplicated images; unreliable data; concerns about the images.

# Molecular Hydrogen Effectively Heals Alkali-Injured Cornea via Suppression of Oxidative Stress

**DOI:** 10.1155/2017/8906027

**Published:** 2017-03-16

**Authors:** Cestmir Cejka, Jan Kossl, Barbora Hermankova, Vladimir Holan, Jitka Cejkova

**Affiliations:** ^1^Institute of Experimental Medicine, Czech Academy of Sciences, 14220 Prague 4, Czech Republic; ^2^Faculty of Natural Science, Charles University, Vinicna 7, 12843 Prague 2, Czech Republic

## Abstract

The aim of this study was to examine the effect of molecular hydrogen (H_2_) on the healing of alkali-injured cornea. The effects of the solution of H_2_ in phosphate buffered saline (PBS) or PBS alone topically applied on the alkali-injured rabbit cornea with 0.25 M NaOH were investigated using immunohistochemical and biochemical methods. Central corneal thickness taken as an index of corneal hydration was measured with an ultrasonic pachymeter. Results show that irrigation of the damaged eyes with H_2_ solution immediately after the injury and then within next five days renewed corneal transparency lost after the injury and reduced corneal hydration increased after the injury to physiological levels within ten days after the injury. In contrast, in injured corneas treated with PBS, the transparency of damaged corneas remained lost and corneal hydration elevated. Later results—on day 20 after the injury—showed that in alkali-injured corneas treated with H_2_ solution the expression of proinflammatory cytokines, peroxynitrite, detected by nitrotyrosine residues (NT), and malondialdehyde (MDA) expressions were very low or absent compared to PBS treated injured corneas, where NT and MDA expressions were present. In conclusion, H_2_ solution favorably influenced corneal healing after alkali injury via suppression of oxidative stress.

## 1. Introduction

Corneal alkali injury often causes extensive damage to the ocular surface and the whole anterior eye segment leading to partial or total vision loss. Immediately after corneal injury, such as alkali burns or irradiation of the cornea with UVB rays, oxidative stress appears in the cornea [1–7]. The activities as well as expressions of corneal antioxidant enzymes substantially decrease, whereas the activities of prooxidant enzymes (e.g., oxidases that generate reactive oxygen species, ROS) remain at physiological levels or even increase. The antioxidant/prooxidant imbalance appears leading to oxidative stress [3]. ROS are insufficiently cleaved. With the effort to substitute the weakened functions of naturally occurring antioxidants, several synthetic antioxidants have been topically applied on the ocular surface with the aim of suppressing oxidative stress and enabling corneal healing [8, 9]. However, Ohta et al. [10] suggested that, despite the clinical importance of oxidative damage, commonly used antioxidants have been of limited therapeutic success. Ohsawa et al. [11] proposed that H_2_ has potential as a novel effective antioxidant in preventive and therapeutic applications. According to these authors H_2_ has a number of advantages as a mild but effective antioxidant: H_2_ rapidly diffuses into tissues and cells, and it is not mild enough either to disturb metabolic redox reactions or to affect ROS that function in cell signaling. H_2_ is an inert gas and only the strong oxidants, for example, hydroxyl radicals and peroxynitrite, are able to oxidize it. In other words H_2_ reacts with strong oxidants such as hydroxyl radical and peroxynitrite in cells, and thus it is a potent agent for preventive and therapeutic antioxidant applications. H_2_ can be consumed in the human body by various ways, including inhaling H_2_, drinking hydrogen water (H_2_-dissolved water), taking a hydrogen bath, injecting H_2_-dissolved saline, dropping H_2_ onto the eye, and increasing the production of intestinal H_2_ by bacteria [10].

Kubota et al. [6] treated corneas burned with alkali (0.15 M NaOH) with various antioxidants, including H_2_. The alkali-injured eyes were irrigated with H_2_ solution of 0.5–0.6 ppm for 30 min. This concentration of H_2_ effectively suppressed oxidative stress in the cornea and reduced corneal neovascularization. The aim of our study was to investigate whether H_2_ solution of similar concentration (0.5–0.6 ppm) would be able to influence the healing of corneas burned with more concentrated alkali (0.25 M NaOH). The injured eyes were irrigated with H_2_ solution (H_2_ in PBS) or PBS free of H_2_ immediately after the injury and then repeatedly for five days. Results show that after H_2_ treatment corneal transparency that was lost after the injury quickly renewed and central corneal thickness that increased after the injury reached physiological levels. On day 20 after the injury in H_2_ treated corneas the intracorneal inflammation was suppressed, the retrocorneal membrane was not developed, and corneal neovascularization was reduced. This was in contrast to PBS treated alkali-injured corneas, where the intracorneal inflammation was highly developed together with the retrocorneal membrane and corneas were largely vascularized.

## 2. Materials and Methods

### 2.1. Preparation of H_2_ Solution in PBS

Original Dr. Hidemitsu Hayashi's Hydrogen Rich Water Stick and original Dr. Hayashi Glass Bottle (The Hydrogen Rich Water Group LLC Lawrence, KS, USA) were employed. The special glass bottle was filled with the PBS and the hydrogen stick was immersed into the bottle. The bottle was tightly closed without the dead volume. The bottle was shaked for 15 sec and left to stand for 45 min. Afterwards the stick was put out from the bottle. The small amount of missing solution was refilled with PBS and the bottle tightly closed.

### 2.2. Measuring H_2_ Concentration in PBS Solution

For the measuring of the concentration of the dissolved molecular hydrogen in PBS (pH 7.2 continually checked by pH meter) the Trustlex ENH-1000 (TRUSTLEX, Kyoto, Japan) was used as the primary measuring device. The Trustlex ENH-1000 is an original Japanese made device for measuring dissolved hydrogen and it displays the dissolved hydrogen by means of hydrogen reduction method in ppm units (wt of H_2_/vol of solution). The measuring method is close to measuring the Oxidative Reduction Potential ORP but this device utilizes an originally developed electrode for detecting the dissolved hydrogen. The device is calibrated directly in ppm (the readings are in ppm).

As a control method for the measuring of molecular hydrogen concentration in PBS buffer the Unisense H_2_ Microsensor was employed. This microsensor is the Clark-type sensor measuring hydrogen partial pressure. The resulting sensor signal is in the pA current range. This signal is measured by the Unisense Microsensor Multimeter. The Multimeter readings can be transferred (according to the manual of the Multimeter) to the concentrations of the dissolved molecular hydrogen in PBS in mmol/L.

The results obtained using both measuring methods differed in 15% of absolute values maximally.

For our experiments (irrigation of eyes) the solution was stored in glass syringes equipped with stop cups. The attention was paid to the fact that no dead volume was present in the syringes. According to Ohta [10] H_2_ can be dissolved in water up to 1.6 ppm, wt/vol (0.8 mM) under atmospheric pressure. In our study the H_2_ concentration measured immediately after preparing the solution was 0.6 ± 0.1 ppm wt/vol. The H_2_ concentration slowly decreased during eye irrigation to the concentration 0.5 ± 0.1 ppm wt/vol on day 5. PBS solution with H_2_ was prepared on the same day when the experiment was started.

### 2.3. Alkali Injury of the Cornea in Experimental Animals

Adult female New Zealand white rabbits (2.5–3.0 kg) were used in our experiments. The investigation was conducted according to the ARVO Statement on the Use of Animals in Ophthalmic and Vision Research. The experiments were approved by the local ethics committee of the Institute of Experimental Medicine under number 11/2013. Rabbits were anesthetized by an intramuscular injection of Rometar (Xylazinum hydrochloricum, Spofa, Prague, CR, 2%, 0.2 mL/kg body weight) and Narkamon (Ketaminum hydrochloricum, Spofa, 5%, 1 mL/kg body weight).

Sodium hydroxide (0.25 M NaOH) was applied by means of dropping on the corneal surface (20 drops during 1 min). Then the eyes (in the first group of animals) were immediately irrigated with H_2_ solution. In the second group of animals the injured eyes were irrigated with PBS. This irrigation of the eyes in both groups lasted 10 min and then the eyes were rinsed with appropriate solutions five times daily (always for two minutes) during five days. Some injured eyes were left without any treatment.

After the alkali injury and awakening from the anesthesia, the rabbits were treated with analgesia (ketoprofen, 1.0 mg/kg i.m.) two times daily for five days. The animals were sacrificed following an i.v. injection of thiopental anesthesia (Thiopental, Spofa, 30 mg/kg) after premedication with an intramuscular injection of Rometar/Narkamon on day 20 after the injury. In all experiments with alkali injury, the corneas of healthy rabbit eyes served as controls. Photographs of the corneas were taken throughout the whole experiment.

### 2.4. Immunohistochemical Examinations

After sacrificing the animals, the eyes were enucleated and the anterior eye segments dissected out and quenched in light petroleum chilled with an acetone-dry ice mixture. Sections were cut on a cryostat and transferred to glass slides. Subsequently, the cryostat sections were fixed in acetone at 4°C for 5 min. For the immunohistochemical detection of Cytokeratin K3/K12, inducible nitric oxide synthase (iNOS), interleukin 1L-*β* (IL-1*β*), *α*-smooth muscle actin (*α*-SMA), nitrotyrosine (NT), malondialdehyde (MDA), and vascular endothelial growth factor (VEGF), the following primary antibodies were used: anti-K3/12 (Abcam, Cambridge, UK), monoclonal mouse anti-iNOS (Biosciences, San Jose, CA, USA), monoclonal mouse anti-NT (Abcam), polyclonal goat anti-MDA (US Biological, Swampscott, MA, USA), mouse monoclonal anti-*α* SMA (Sigma, Saint Louis, MO, USA), anti-IL-1*β* (Thermo Fisher Scientific, https://www.thermofisher.com/cz/en/home/life-science/antibodies.html), and mouse monoclonal anti-VEGF (Abcam). The binding of the primary antibodies was demonstrated using the HRP/DAB Ultra Vision detection system (Thermo Scientific, Fremont, CA) following the instructions of the manufacturer: hydrogen peroxide block (15 min), ultra V block (5 min), primary antibody incubation (60 min), biotinylated goat anti-mouse IgG (Lab Vision, Fremont, CA), or donkey anti-goat IgG (Santa Cruz Biotechnology) secondary antibody incubation (10 min) and peroxidase-labeled streptavidin incubation (10 min). Visualization was performed using a freshly prepared DAB substrate-chromogen solution. Cryostat sections in which the primary antibodies were omitted from the incubation media served as negative controls. Sections were counterstained with Mayer's hematoxylin.

### 2.5. Determination of Corneal Thickness

Changes of corneal optical properties after the injury and during healing were evaluated by measuring the central corneal thickness (taken as an index of corneal hydration) (see [12] in detail). Briefly, the central corneal thickness was measured in anesthetized animals using an ultrasonic pachymeter SP-100 (Tomey Corporation, Nagoya, Japan) in the corneal center. The corneal thickness was measured in the same corneas before alkali injury (corneas of healthy eyes) and two, five, ten, and twenty days after the injury (all experimental groups). Each cornea was measured four times and the mean value and standard deviation of the thickness (in *μ*m) were computed.

### 2.6. Evaluation of Corneal Neovascularization and Transparency

For evaluation of corneal neovascularization, the number of vessels was counted in each of 60° sectors of the corneal surface. The mean value and standard deviation were counted from five measurements. This procedure was applied for every eye from a matching group of eyes (control, injured, and treated with H_2_ solution and injured and treated with buffer).

### 2.7. Detection of Gene Expression by Real-Time PCR

The expression of genes for K3, K12, IL-1*β*, and VEGF in control and treated corneas was determined by quantitative real-time polymerase chain reaction (PCR). Corneas were excised using Vannas scissors, transferred into Eppendorf tubes, and immediately frozen. The frozen corneal tissue was then homogenized and added in 500 *μ*L of TRI Reagent (Molecular Research Center, Cincinnati, OH) for the RNA isolation. The details of RNA isolation, transcription, and the PCR parameters have been described previously [13]. In brief, total RNA was extracted using TRI Reagent according to the manufacturer's instructions. One *μ*g of total RNA was treated using deoxyribonuclease I (Promega) and subsequently used for reverse transcription. The first-strand cDNA was synthesized using random primers (Promega, Madison, WI) in a total reaction volume of 25 *μ*L, using M-MLV Reverse Transcriptase (Promega). Quantitative real-time PCR was performed in a StepOnePlus real-time PCR system (Applied Biosystems). The relative quantification model with efficiency correction was applied to calculate the expression of the target gene in comparison with GAPDH used as the housekeeping gene. The following primers were used for amplification: GAPDH: 5′-CCCAACGTGTCTGTCGTG (sense), 5′- CCGACCCAGACGTACAGC (antisense), K3: 5′′-GAACAAGGTCCTGGAGACCA (sense), 5′-TTGAAGTCCTCCACCAGGTC (antisense); K12: 5′′-AGGAGGTGGTGAATGGTGAG (sense), 5′-GTTGTTTCCCAGGAGCAAAA (antisense). IL-1*β* 5′-CTGCGGCAGAAAGCAGTT (sense), 5′- GAAAGTTCTCAGGCCGTCAT (antisense) and VEGF: 5′-CGAGACCTTGGTGGACATCT (sense), 5′-ATCTGCATGGTGACGTTGAA (antisense). The PCR parameters included denaturation at 95°C for 3 min, then 40 cycles at 95°C for 20 s, annealing at 60°C for 30 s, and elongation at 72°C for 30 s. Fluorescence data were collected at each cycle after an elongation step at 80°C for 5 s and were analyzed on the StepOne Software, version 2.2.2 (Applied Biosystems). Each individual experiment was done in triplicate. In figure legends each bar represents the mean ± SD from 6 individual corneas. In Figure 1 the value of control corneas for K3 and K12 is taken as 100% corresponding to the values of relative gene expression 18800 for K3 and 1750 for K12. In Figure 2 the value of control corneas for IL-1*β* is taken as 100% corresponding to the value of relative gene expression 120. In Figure 5 the value of control corneas for VEGF is taken as 100% corresponding to the value of relative gene expression 440.

### 2.8. Statistics

An analysis of the data showed normal distribution and the results are expressed as mean ± SD. Comparisons between the two groups were made by Student's *t*-test, and multiple comparisons were analyzed by ANOVA. A value of *P* < 0.05 was considered statistically significant.

## 3. Results

In our study, besides two groups of corneas, alkali-injured treated with H_2_ solution or with PBS, there was the group of animals, which were left without any treatment after the injury was used. Furthermore, the alkali-injured group of corneas was treated with PBS after purge of H_2_ used as a negative control. Because immunohistochemical, biochemical, and macroscopical results and results obtained with ultrasonic pachymeter of injured untreated corneas and corneas treated with PBS after purge of H_2_ did not significantly differ from results obtained with injured corneas treated with PBS, we did not show the results with injured untreated group and group treated with PBS after purge of H_2_.

### 3.1. Immunohistochemical Detection of K3/K12, iNOS, IL-1*β*, *α*-SMA, VEGF, and Gene Expression of K3, K12, IL-1*β*, and VEGF in Control Healthy Corneas and in Injured Corneas Treated with H_2_ Solution or PBS (Day 20 after the Injury)

The expressions of K3/K12 were high in injured corneas treated with H_2_ solution (Figure 1(c)) (compared with control cornea, Figure 1(d)), whereas the expressions were low in corneas treated with PBS (Figure 1(b)), where only flat epithelium was present (Figure 1(d)). Some corneas were without epithelium (Figure 1(a)). The expression of genes for K3 and K12 in control (healthy), injured PBS treated, and injured corneas treated with H_2_ solution was quantified by real-time PCR (Figures 1(e) and 1(f)). The treatment of injured corneas with H_2_ solution significantly increased the expression of K3 and K12. The expression of iNOS and IL-1*β* was high in injured corneas treated with PBS (Figures 2(a) and 2(b)), whereas they were low or absent in injured corneas treated with H_2_ solution (Figures 2(c) and 2(d)), similarly to in control corneas (Figures 2(e) and 2(f)). The expression of genes for IL-1*β* (Figure 2(g)) in control (healthy), injured PBS treated, and injured corneas treated with H_2_ solution was quantified by real-time PCR. The expressions of NT and MDA were not present in injured corneas treated with H_2_ solution (Figures 3(c) and 3(d)), whereas the expressions of NT and MDA were high in injured PBS treated corneas (Figures 3(a) and 3(b)) compared to control corneas, where the expressions of NT and MDA were absent (Figures 3(e) and 3(f)). The expression of *α*-SMA was high in the corneal stroma of injured PBS treated corneas (Figure 4(a)) and in retrocorneal membrane (Figure 4(b)). In injured corneas treated with H_2_ solution, *α*-SMA was very low in the corneal stroma (Figure 4(c)) and the retrocorneal membrane was not developed (Figure 4(d)), similarly as in control cornea (Figures 4(e) and 4(f)). The expression of gene for VEGF was high in injured PBS treated corneas (Figure 5(a)) and nearly absent in injured corneas treated with H_2_ solution (Figure 5(b)). In control corneas (Figure 5(c)) VEGF expression was absent. The expression of gene for VEGF in control (healthy), injured PBS treated, and injured corneas treated with H_2_ solution was quantified by real-time PCR (Figure 5(d)).

### 3.2. Corneal Opacity and Neovascularization of Alkali-Injured Eyes Treated with H_2_ Solution or PBS

Representative photographs of healthy and injured eyes treated with H_2_ solution or PBS are shown in Figure 6. In comparison with the healthy control eyes (Figure 6(a)), corneas of injured eyes became opalescent immediately after the injury (Figure 6(b)). Following PBS treatment the injured corneas remained opalescent until day 20 and in the last days the corneas were vascularized. This was in contrast to H_2_ solution treated corneas, where the corneal transparency was renewed during five days after the injury and corneal neovascularization was highly suppressed until day 20.

### 3.3. Central Corneal Thickness after Alkali Injury and Treatment with H_2_ Solution or PBS

Shortly after alkali injury, the central corneal thickness increased more than twice (compared to levels before injury, day 0) and in PBS treated injured corneas remained elevated until day 20 after the injury. In H_2_ solution treated corneas the central corneal thickness was reduced from day two to day five and on day 10 the corneal thickness returned to the values before injury (day 0) (Figure 7(a)). Quantification of corneal neovascularization is summarized in Figure 7(b).

## 4. Discussion

In chemical corneal burns, such as burning of the cornea with sodium hydroxide, alkali quickly penetrates through the cornea into the inner eye damaging tissues and therefore the emergency intervention and the early effective therapy are necessary for vision restoration. H_2_ proved to be suitable for these purposes. H_2_ has no cytotoxicity even at high concentration [10]. It quickly penetrates through tissues and cells and suppresses oxidative stress occurring in the anterior eye segment immediately after the injury, such as alkali burns or UVB irradiation [1–7]. After corneal injuries, the imbalance between antioxidants and prooxidants appeared in the cornea, resulting in oxidative stress. Wakamatsu et al. [14] described that an imbalance between free radical-generating and radical-scavenging systems resulting in oxidative stress represents a condition that has been associated with the cell injury seen in many pathological states. According to these authors, the effects of ROS are wide-ranging, but three reactions are particularly relevant to cell injury: lipid peroxidation of membranes, oxidative modification of proteins, and oxidative damage to DNA. Our results show that the treatment of alkali-injured corneas with H_2_ solution highly suppressed oxidative stress in the cornea, resulting in favorable corneal healing. During 10 days after the injury with alkali and repeated irrigation of injured eyes with H_2_ solution, corneal transparency—lost after the injury—highly restored (Figure 6) and central corneal thickness (corneal hydration)—increased after the injury—achieved before injury levels (Figure 7). Later (on day 20 after the injury), in alkali-injured corneas treated with H_2_ solution, the expressions of NT and MDA were low or absent, whereas in PBS treated injured corneas NT and MDA expressions were present (Figure 3). It is suggested that H_2_ quickly penetrating into the cornea after the dropping onto the damaged ocular surface effectively prevented or highly suppressed peroxynitrite formation and lipid peroxidation in the cornea. According to Ohsawa et al. [11] H_2_ cleaves the hydroxyl radicals thus preventing subsequent lipid peroxidation, DNA oxidation, and mitochondrial dysfunction. According to these authors inhalation of H_2_ in a rat model of cerebral ischemia-reperfusion injury effectively reduced ROS-induced brain damage. Ohta [10] described that H_2_ shows not only effects against oxidative stress, but also various anti-inflammatory and antiallergic effects. In our study H_2_ solution significantly suppressed intracorneal inflammation (Figure 2).

The alkali-injured corneas treated with PBS healed with fibrosis and scarring. In these corneas high expressions of *α*-SMA (a marker of myofibroblasts) were present (Figure 4). Myofibroblasts differentiate from stromal keratocytes in the vicinity of the wound [15]. Myofibroblasts are necessary for corneal healing; however, their accumulation and persistence in injured areas is associated with corneal scarring [16]. Myofibroblasts produce the anomalous extracellular matrix which contributes to corneal opacity [17]. In our study, in alkali-injured corneas treated with H_2_ solution, damaged corneas healed with the restored corneal transparency (Figure 6). In the injured part of the corneal stroma the expression of *α*-SMA was reduced (Figure 4). Myofibroblasts expressing high levels of *α*-SMA [18–20] are modulated by proinflammatory cytokines, such as IL-6 and IL-1*β* [17, 21]. In our study, in injured corneas treated with H_2_ solution the levels of IL-1*β* were reduced (Figure 2). This is in accordance with previous papers in which significant suppression of proinflammatory cytokines and oxidative stress injury after H_2_ therapy was described in various diseased tissues and organs (e.g., [22]).

Myofibroblasts produce nitric oxide by iNOS in response to cytokine stimulation [23]. Besides myofibroblasts also corneal cells and inflammatory cells express iNOS in diseased corneas [24]. This is in accordance with our findings. High expressions of iNOS were present in PBS treated alkali-injured corneas, whereas in injured corneas treated with H_2_ iNOS expression was significantly reduced or completely absent (Figure 2).

The development of retrocorneal membrane after the injury with more concentrated alkali seriously threatens vision [18]. During healing of damaged alkali-injured corneas, the fibrous structure is formed in the endothelial layer beneath Descemet's membrane [25]. According to these authors, during fibrogenic reaction, corneal endothelial cells undergo mesenchymal transition and transform to myofibroblasts. In this study, the retrocorneal membrane was formed in PBS treated alkali-injured corneas and it was absent in injured corneas treated with H_2_ solution (Figure 4).

## 5. Conclusions

The treatment of alkali-injured corneas with H_2_ solution favorably influenced corneal healing via antioxidant and antiinflammatory effects. As found previously [10, 26], H_2_ selectively reduces strong oxidants, such as hydroxyl radicals and peroxynitrite, and exhibits cytoprotective effects against oxidative stress [11]. Kubota et al. [6] found that H_2_ therapy of the cornea burned with lower concentration of alkali (0.15 M NaOH) reduced ROS production in the cornea and corneal neovascularization. We investigated in this study that H_2_ solution effectively suppressed oxidative stress in the cornea and decreased corneal neovascularization, even if the cornea was burned with higher concentrated alkali (0.25 M NaOH). After H_2_ treatment peroxynitrite, a product from the reaction of superoxide with nitric oxide, was reduced and formation of MDA was prevented or decreased. MDA serves as a marker of oxidative stress [27]. Furthermore, H_2_ prevented formation of retrocorneal membrane, feared complication of corneal alkali burns, making residual vision impossible. Injured corneas treated with H_2_ solution healed with the renewal of corneal transparency without scarring and neovascularization. H_2_ has a potent antiscarring effect. Because H_2_ is therapeutically very effective and simultaneously nontoxic and nonfunctional in human cells [10], it can be employed separately for the treatment of various ocular disorders or in combination with other required therapy. In conclusion, H2 therapy of the anterior eye segment after alkali burns of the cornea was effective for vision restoration similarly as H_2_ therapy of the posterior eye segment diseases described previously [28–30].

## Figures and Tables

**Figure 1:** The immunohistochemical detection of cytokeratins K3/K12 and the expression of genes for cytokeratins K3 (e) and K12 (f) determined by real-time PCR in injured corneas treated with H_2_ dissolved in PBS (H_2_) or with PBS free of H_2_ (buffer) examined on day 20 after the injury. The expression of K3/K12 was high in injured reepithelialized corneas treated with H_2_ (c), arrow points to the epithelium, whereas in injured corneas treated with buffer, where corneas were poorly reepithelialized (arrows), the expressions of K3/K12 were low or absent (a, b) compared to the control cornea (d). Scale bars: 50 *μ*m. In graphs the values with asterisks represent statistically significant (^*∗∗∗*^*P* < 0.001) difference from injured buffer treated corneas.

**Figure 2:** The immunohistochemical detection of iNOS and IL-1*β* and the expression of genes for IL-1*β* (g) determined by real-time PCR in injured corneas treated with H_2_ dissolved in PBS (H_2_) or with PBS free of H_2_ (buffer) examined on day 20 after the injury. The expressions of iNOS (a) and IL-1*β* (b) were high in buffer treated injured corneas, arrows, whereas in H_2_ treated injured corneas the expressions of iNOS (c) and IL-1*β* (d) were low or completely absent, similarly to in control cornea for iNOS (e) or IL-1*β* (f). Scale bars: 50 *μ*m. In graph the values with asterisks represent statistically significant (^*∗∗∗*^*P* < 0.001) difference from injured buffer treated corneas.

**Figure 3:** The immunohistochemical detection of nitrotyrosine (NT) and malondialdehyde (MDA) in injured corneas treated with H_2_ dissolved in PBS (H_2_) or with PBS free of H_2_ (buffer) examined on day 20 after the injury. In buffer treated injured corneas the expressions of NT (a) and MDA (b) were high (arrows). This was in contrast to H_2_ solution treated injured corneas, where the expressions of NT (c) and MDA (d) were absent, similarly to in control corneas (e, f). Scale bars: 50 *μ*m.

**Figure 4:** The immunohistochemical detection of *α*-SMA in injured corneas treated with H_2_ dissolved in PBS (H_2_) or with PBS free of H_2_ (buffer) examined on day 20 after the injury. The expression of *α*-SMA was high in the corneal stroma of injured corneas treated with buffer (a) (arrow) and in retrocorneal membrane (arrow) (b), whereas in injured corneas treated with H_2_ the expression of *α*-SMA was low in the corneal stroma (c) and the retrocorneal membrane was not developed (d) compared to control cornea (e, f). Scale bars: 50 *μ*m.

**Figure 5:** The immunohistochemical detection of vascular endothelial growth factor (VEGF) in injured corneas treated with H_2_ dissolved in PBS (H_2_) or with PBS free of H_2_ (buffer) examined on day 20 after the injury. In buffer treated corneas the expression of VEGF was high (a), (arrows) and corneas are vascularized, whereas the expression of VEGF in damaged corneas after H_2_ treatment was low (b) compared with control cornea (c). Scale bars: 50 *μ*m. The expression of genes for VEGF determined by real-time PCR (d). In graphs the values with asterisks represent statistically significant (^*∗∗*^*P* < 0.01) difference from injured buffer treated corneas.

**Figure 6:** Corneal opacity of alkali-injured eye and injured eyes treated with H_2_ dissolved in PBS (H_2_) or with PBS free of H_2_ (buffer). Representative photographs show control healthy eye (a), alkali-injured eye (immediately after the injury) (b), the injured eye treated with H_2_ solution from day 2 to day 20 (c, d, e, f), and injured eye treated with buffer from day 2 to day 20 (g, h, i, j). Corneal transparency renewed only in corneas treated with H_2_ solution. Corneas treated with buffer remained opalescent and corneas were vascularized. Arrows point to vessels.

**Figure 7:** Central corneal thickness of control (healthy) cornea and alkali-injured corneas treated with H_2_ dissolved in PBS (H_2_) or with PBS free of H_2_ (buffer) (a). Central corneal thickness was measured in the same rabbit before injury (day 0) and on days 2, 5, 10, and 20 after the injury. In buffer treated injured corneas and in H_2_ solution treated injured corneas the values for days 2 and 5 are statistically different (^*∗∗*^*P* < 0.01, ^*∗∗∗*^*P* < 0.001) from the values before injury. In H_2_ treated injured corneas the values for days 10 and 20 are not significantly different (n.s.) from values before injury. This is in contrast to buffer treated injured corneas, where the values for days 10 and 20 remain statistically different (^*∗*^*P* < 0.05, ^*∗∗∗*^*P* < 0.001) from values before injury. The quantification of corneal neovascularization is shown in (b). The number of vessels was high in buffer treated injured corneas and was significantly reduced in injured corneas treated with H_2_. The values with asterisks are significantly different (^*∗∗∗*^*P* < 0.001) from values with buffer treated injured corneas.

## Abbreviations

ROS: Reactive oxygen species
NT: Nitrotyrosine
MDA: Malondialdehyde
K3, K12: Cytokeratins K3, K12
IL-1*β*: Interleukin-1*β*
IL- 6: Interleukin-6
iNOS: Inducible nitric oxide synthase
*α*-SMA: *α* smooth muscle actin
TGF-*β*1: Transforming growth factor-beta 1
VEGF: Vascular endothelial growth factor.

## Additional Points

*Highlights*. Alkali induces corneal damage causing vision impairment. In alkali-injured cornea oxidative stress appears. The antioxidant/prooxidant imbalance results in oxidative stress. Suppression of oxidative stress by H_2_ treatment leads to favorable corneal healing.
